# The Relationship between Physical Activity and Health-Related Quality of Life (HINT-Eight) in Middle-Aged Korean Women

**DOI:** 10.1155/2022/4555547

**Published:** 2022-10-04

**Authors:** Myung-Nam Lee, Sang-Dol Kim, Young-Soon Choi

**Affiliations:** Department of Nursing, Kangwon National University, Samcheck-si, Gangwon-Do 25949, Republic of Korea

## Abstract

The purpose of this study was to provide basic data on health by examining the effect of HINT-eight on the physical activity of middle-aged Korean women using secondary data from the 2019 KNHANES. The subjects were 1,428 middle-aged women aged 45-64. Multiple regression was performed to verify the relationship between physical activity and HINT-eight. Following confirmation of the association between HINT-eight and physical activity, it was found that the subdomains of QOL, such as stair climbing, vitality, work, sleeping, and happiness, were connected to physical activity. Stair climbing positively affected physical activity, education level, and grip strength and negatively affected age. Pain positively affected education level and grip strength and negatively affected age. Vitality positively affected physical activity, monthly household income, and grip strength. Working positively affected education level, monthly household income, and grip strength and negatively affected age. Depression positively affected monthly household income. Memory and sleep positively affected education level and negative effect on age. Happiness positively affected physical activity and monthly household income. In this study, physical activity was found to have an effect on various factors of QOL. Physical activity in middle age is an important influencing factor on the QOL in old age; to improve the QOL in older adult, it is necessary to make efforts to improve physical activity in middle age.

## 1. Introduction

Middle-aged women are defined by the complex interaction of environmental and psychological factors, and they may be classified as middle-aged women who connect a stable life process from adulthood to just before the onset of old age [1]. Since the definition of the middle-aged class is different for each scholar, it is not easy to distinguish them academically. Middle-aged was defined as a woman between the ages of 45 and 64, who showed a tendency toward menopause and aging due to physical decline in all organs and hormonal changes, and was sensitive to physical changes [2]. Middle-aged is a physiological transition period for women to experience various physical and mental health problems and various syndromes due to menopause [3]. During that time, middle-aged women face a loss in physiological functioning, aging, and menopause and obesity and body imbalances owing to an increase in body weight and abdominal fat. In addition, a decrease in bone density in the bone causes osteoporosis and fractures. Hormonal changes due to imbalance of the endocrine system and ataxia of the autonomic nervous system due to mental stress cause symptoms such as fever, sweating, chills, dull sensation, cold hands and feet, palpitations, and headaches [3]. Moreover, weakness, fatigue, dizziness, and syncope appear irregularly, and atrophic cystitis and urinary incontinence due to degenerative changes in the genitourinary system occur frequently. Following physical health issues, individuals may endure emotional issues such as depression, loneliness, and feelings of failure [3]. Middle-aged women are reported to have higher morbidity than men in inducing health problems due to neglect of health care because role conflicts and various life events are affecting their psychological adaptation ability due to psychological and social role changes [4]. Furthermore, antioxidant enzyme activity and aging are known to be intimately associated because the rapid loss in antioxidant enzymes with age reduces the ability to respond to free radicals or lipid peroxides, and the organs and cells gradually diminish [5]. Obesity, which is one of the causes of various diseases, is caused by the influence of lack of physical activity or excessive intake and genetic factors. It also refers to a condition in which the body accumulates an excess of fat as a result of an imbalance between the amount of energy used and the amount of energy consumed [6]. This can be addressed by increasing physical activity.

Regular exercise is the best way to prevent diseases by preventing an increase in body fat percentage and a decrease in muscle mass in middle-aged and by activating the energy metabolism function of the muscles. Accordingly, interest in the necessity of exercise therapy and specific methods is gradually increasing [7]. Despite the scientific and empirical recognition that regular exercise for middle-aged women can improve their health, 63.1% of middle-aged women do not exercise regularly [8]. Among these health promotion activities performed by middle-aged women, the exercise area has the lowest practice rate [9]. Therefore, it is important to identify the factors affecting the quality of life (QOL) of physical activity to increase the practice of physical activity among middle-aged women. For many years, exercise and physical activity has been proposed as a treatment option and has attracted the attention of researchers and clinicians [10, 11]. Studies have shown that more moderate exercise habits are correlated with lower levels of depressive symptoms and higher levels of mental health [12, 13], appearing to improve QOL.

The purpose of this study is to provide basic data on health by examining the effects of physical activity on health-related quality of life (HINT-eight) in middle-aged Korean women. The specific goals are as follows. Check the difference between the general characteristics and HINT-eight according to physical activity. Check the relationship between physical activity and HINT-eight and identify the factors affecting HINT-eight.

## 2. Theoretical Background

Physical activity refers to any movement of the body that result in a significant increase in energy expenditure through the contraction of skeletal muscles in everyday life; including regular exercise that demands energy consumption above a steady state [14, 15]. It has been reported that a decrease in physical activity lowers the level of muscle strength and cardiopulmonary function, thereby increasing the incidence of metabolic syndrome and affecting the incidence of adult diseases such as hypertension and diabetes [16]. The word aerobic exercise means that energy was produced using oxygen during exercise. Aerobic exercise maintains human life by continuously taking in oxygen from the body, and when it stimulates the activity of the heart and lungs, it has the effect of strengthening blood vessels and facilitating all functions in the body normally [17]. According to the guidelines of the recommended guidelines for physical activity recommended by the World Health Organization (WHO) [18], at least 150 minutes per week of moderate-intensity aerobic exercise or 75 minutes or more of vigorous-intensity aerobic exercise is recommended for a healthy life [19]. Aerobic exercise effectively improves the risk of arteriosclerosis and blood lipids, and it is essential for preventing obesity-related diseases by boosting energy metabolism with fat to inhibit and utilize fat tissue buildup caused by obesity. The composition of aerobic exercise can be configured to improve cardiorespiratory function and increase maximum oxygen intake [19].

Physical activity through exercise is a safe and cost-effective technique for lowering blood pressure and other cardiovascular and metabolic diseases. In particular, the postexercise hypotension (PEH) response that appears in the recovery period after exercise is a phenomenon in which blood pressure continues to decrease after a one-time exercise. It is expressed in a complex way under the influence of environmental factors along with various neurological and hemodynamic changes such as baroreflex regulation, decreased sympathetic nerve activity, increased vasodilation, decreased vascular resistance, and fluid regulation [20]. Various studies have shown that exercise and physical activity can reduce somatic symptoms, for example, by improving sleep [21] and sexual function [22]. Reducing affective and cognitive symptoms can also be achieved by reducing stress [23], improving and expanding coping methods [24], and increasing positive emotions [25]. Accordingly, it seems that exercise and physical activity can improve affective by enhancing positive emotions [26].

Health management is the most important thing in extending the life facing, and in modern life, weight gain and loss of physical strength are progressing due to lack of exercise. Therefore, it is necessary for middle-aged women to promote health through active physical activities such as exercise and sports [27]. As interest in obesity expands, studies are being reported that regular exercise can reduce obesity. Obesity can be overcome by engaging in moderate-intensity physical activity at least three times per week for at least 30 minutes each day [28]. Recently, in evaluating an individual's health, it is not simply a disease-free state, but rather an individual's physical health, social and psychological functions, and overall health including role are emphasized [29]. When considered as representing the degree of human well-being and well-being, QOL is a subjective value assessment that an individual feels in everyday life and is represented as life satisfaction or happiness [30].

Although it is not easy for middle-aged women to adapt physically, mentally, and socially, it can depend on how they accept their changes [31]. The QOL of middle-aged women can be said to be the degree of subjective satisfaction experienced in relation to menopausal symptoms. Therefore, the more the symptoms of menopause are experienced and severe, the longer the QOL decreases, and therefore, the more experienced the more severe, and the longer the menopausal symptoms, the lower the QOL [31]. As a result, middle-aged women are experiencing quick and diversified psychological changes, which can be viewed as a crisis in terms of health management, whereas health promotion habits in other areas are being adopted relatively [9]. Therefore, it is reported that middle-aged women who are in a crisis of health undergo rapid changes, even though it is a time when health promotion should be specially emphasized, while the exercise practice rate is reported to be quite low. In the middle-aged, when the prevalence of various health problems and chronic diseases is increasing, it is important to maintain and promote health through daily life to secure a healthy lifespan [9].

In Korea, there have been few cases in which HRQOL tools for the general population have been developed, and the tools developed in the past National Health and Nutrition Examination Survey had a large number of items, so it was difficult to use them for the entire population. In addition, in the case of tools developed abroad, there may be limitations in sufficiently reflecting the HRQOL of Koreans, so HINT-8 was developed [32]. Indirect measurement tools for measuring HRQOL include EQ-five D, SF-36, and HUI. As direct measurement tools, EQ-VAS (Visual Analog Scale), Standard gamble, and Time trade-off are used. Among them, EQ-five D-three L has the advantage of simple questions and short survey time, so it is widely used as a national survey tool such as the National Health and Nutrition Examination Survey, Community Health Survey, and Korea Medical Panel Survey [23, 32, 33]. However, EQ-five D is a tool developed in Europe, suggesting that EQ-five D may not reflect the unique characteristics of each country [32, 34]. Korean Health-related Quality of Life Instrument with eight items (HINT-eight) was developed with the goal of more accurately measuring health-related quality of life (HRQOL) suitable for the characteristics of Koreans. It consists of four domains (physical health domain, social health domain, mental health domain, and positive health domain) and detailed items (stair climbing, pain, vitality, work, depression, memory, sleeping, and happiness). There are four level questions for each item, so the number of health conditions that can be expressed is 65,536, which is much richer than the 3,125 of EQ-five D-five L. In addition, because of a HINT-eight questionnaire survey to 892 adults nationwide, 12.3% answered that there was no problem in all items, which showed that the ceiling effect was lower than that of EQ-five D-five L (76.3%). This means that HINT-eight can show the HRQOL of the public in Korea more precisely than the EQ-five D tool [32, 34].

Despite the advantages of HINT-eight, this tool has not been developed for a while, and follow-up studies have not been conducted properly, so its utility is insignificant so far [23]. Therefore, in this study, HINT-eight was used to analyze HRQOL according to physical activity and to use it as data to improve the QOL of middle-aged women.

## 3. Research Method

### 3.1. Study Design

This study is a cross-sectional descriptive research study to confirm the effect of physical activity on QOL in middle-aged women. The data used are open public secondary data from the National Health and Nutrition Examination Survey (KNHANES) conducted by the Korea Centers for Disease Control and Prevention (KCDC), and the QOL related to health according to physical activity was confirmed using the basic data (Approval No. 117002) [35].

### 3.2. Participants and Procedure

This study used data from the eighth KNHANES conducted in 2019. The KNHANES is a survey on health behavior, prevalence of chronic diseases, food, and nutrition conducted under Article 16 of the National Health Promotion Act. In addition, it is an open public statistical data designated by the Korean government in accordance with Article 17 of the Statistical Act (Approval No. 117002). The KNHANES is a nationwide health and nutrition examination survey conducted by the Korean Ministry of Health and Welfare and the KCDC, with the aim of producing representative and reliable statistics on national and municipal scales regarding the health status, health behavior, and nutrition status of the Korean people. Sampling bias was controlled through sampling guidelines in the KCDC to which clustered, multistage, stratified, and probability sampling was applied [35].

Prior to data collection, informed consent was obtained from all study participants, and data collection was performed by the KCDC in compliance with research ethics guidelines [35]. The data can be used for research purposes alone, can only be accessed in accordance with the KCDC guidelines, and do not contain information that can identify individual participants. Among the effective sample of 8,110 people in the total sample, 1,428 middle-aged women aged 45-64 years were collected as data through case selection. The survey of this data was conducted in a circular stratified sampling method from January-December 2019. This data was investigated using the health survey method, such as household survey, health interview survey, and health behavior survey (self-reported survey) [35].

### 3.3. Research Tools

#### 3.3.1. Physical Activity

In this study, the practice of physical activity refers to the practice of physical activity in the data of the KNHANES. Physical activity means engaging in moderate-intensity physical activity for at least 2 hours and 30 minutes per week, or engaging in high-intensity physical activity for at least 1 hour and 15 minutes, or it is a combination of moderate-intensity and high-intensity physical activity (1 minute of high‐intensity physical activity = 2 minutes of moderate‐intensity physical activity). High-intensity physical activity refers to vigorous physical activity that results in shortness of breath or a very fast heartbeat, and “moderate physical activity” refers to moderate-intensity physical activity that results in slightly shortness of breath or slightly rapid heartbeat [35].

#### 3.3.2. Health-Related Quality of Life (HRQOL)

The HRQOL in this study was measured with the Korean Health-related Quality of Life Instrument with eight items (HINT-eight) of the KNHANES data designed to discriminate healthy population groups [32, 35]. The physical health domain of HINT-eight-four L consists of three subfactors: stair climbing, pain, and vitality. The questions measuring the stair climbing factor were designed with questions such as “1 = I had no difficulty climbing stairs, 2 = I had some difficulty climbing stairs, 3 = I had a lot of difficulties climbing stairs, and 4 = I could not climb stairs.” The questions measuring the pain factors were designed with questions such as “1 = I had no pain at all, 2 = I had mild pain, 3 = I had severe pain, and 4 = I had extreme pain.” The questions to measure the vitality factor were designed such as “1 = I was always energetic, 2 = I was often energetic, 3 = I was occasionally energetic, and 4 = I was not energetic at all.” The social health domain of HINT-eight-four L is composed of work factors. The questions measuring the work factors were designed with questions such as “1 = I had no difficulty at work, 2 = I had some difficulty at work, 3 = I had a lot of difficulty at work, and 4 = I could not work.” The mental health domain of HINT-eight-four L consists of three subfactors: depression, memory, and sleep. The questions measuring the depressive factors were designed such as “1 = I was never depressed, 2 = I was sometimes depressed, 3 = I was often depressed, and 4 = I was always depressed.” The questions measuring the memory factors were designed such as “1 = I had no difficulty remembering at all, 2 = I had some difficulty remembering, 3 = I had a lot of difficulties remembering, and 4 = I had no memory at all.” The questions measuring the sleep factors were designed such as “1 = I had no difficulty falling asleep, 2 = I had some difficulty sleeping, 3 = I had a lot of trouble falling asleep, and 4 = I could not sleep.” The positive health domain of HINT-eight-four L consists of happiness factors. The questions measuring the happiness factor were designed with questions such as “1 = I was always happy, 2 = I was often happy, 3 = I was sometimes happy, and 4 = I was not happy at all” [32, 35].

### 3.4. Data Analysis Method

The data collected in this study were using the SPSS 21.0 program. Frequency and percentage were conducted to find out the demographic characteristics. A *χ*^2^-test was conducted to confirm the relationship between demographic characteristics, health status, health behavior, physical variables, and presence or absence of physical activity. The correlation between physical activity and eight subfactors of HINT-eight-four L were analyzed by Pearson's correlation; factors affecting HINT-eight-four L were identified by multiple regression analysis.

## 4. Research Results

### 4.1. Difference in Physical Activity according to General Characteristics

Table 1 shows the differences in physical activity according to general characteristics. As a result of a survey of 1,428 people to confirm the relationship between the subject's characteristics and physical activity, age and physical activity were found to be correlated with each other (*x*^2^ = 7.057, *p* < 0.05). 11.5% in their 40s, 21.0% in their 50s, and 9.0% in their 60s were found to engage in physical activity. There was no correlation between marital status and physical activity. 33.3% living together, 4.4% separated or divorced, 2.6% widowed, and 1.1% single were found to engage in physical activity. Educational level and physical activity were found to be correlated with each other (*x*^2^ = 11.008, *p* < 0.01). It was found that 4.0% of elementary school graduates or less, 4.7% of middle school graduates, 19.3% of high school graduates, and 13.5% of college graduates or higher engage in physical activity. The residential area and physical activity were found to be correlated (21,*p* < 0.001). It was found that 6.0% of eup and myeon residents and 35.4% of dong residents engaged in physical activity.

### 4.2. Relationship between Subjects' HINT-Eight and Physical Activity

Because of confirming the relationship between the subject's quality of life related to health (HINT-8) and physical activity, the results shown in Table 2 were obtained. The relationship between stair climbing and physical activity was found to be statistically significant (*x*^2^ = 23.964, *p* < 0.001). As for the responses of the subjects, it was found that 23.4% of the subjects had no difficulty climbing stairs, 16.9% had some difficulty, and 1.2% had a lot of difficulty doing s physical activity. The relationship between pain and physical activity was not statistically significant. As for the responses of the subjects, no pain at all 16.0%, slightly present 22.3%, severe pain 2.7%, and excruciating pain 0.5% were found to be physical activity. The correlation between vitality and physical activity was found to be statistically significant (*x*^2^ = 20.452, *p* < 0.001). The subjects' vitality was always present 14.0%, frequently 14.5%, occasionally 12.3%, and never at all 0.8% showed physical activity. The relationship between work and physical activity was found to need further confirmation statistically (*x*^2^ = 6.501, *p* < 0.10). It was found that 23.5% of the subjects had no difficulty working at all, 16.1% had a little, 1.5% had a lot, and 0.4% could not do physical activity. The relationship between depression and physical activity was not statistically significant. 20.7% were not depressed at all, 19.0% were occasionally depressed, 1.5% were often depressed, and 0.3% always depressed were found to engage in physical activity. The correlation between memory and physical activity was not statistically significant. There was no difficulty in remembering at all = 17.1%, a little bit = 23.5%, and a lot = 0.9% showing physical activity. The relationship between sleep and physical activity was found to be statistically significant (*x*^2^ = 7.049. *p* < 0.01). 18.7% had no difficulty sleeping at all, 23.5% had a little, 4.0% had a lot, and 0.3% had difficulty sleeping. The relationship between happiness and physical activity was found to be statistically significant (*x*^2^ = 13.300, *p* < 0.01). Always happy = 8.3%, often happy = 17.5%, occasionally happy = 14.4%, and never happy = 1.4% were found to engage in physical activity.

### 4.3. Correlation between HINT-Eight and Physical Activity

The correlation between the subject's physical activity and HINT-eight is as follows [Table 3]: Physical activity showed a positive correlation with stair climbing (*r* = .095, <.001), vitality (*r* = .095, *p* < .001), and happiness (*r* = .072, *p* < .001). Stair climbing showed a positive correlation with pain (*r* = .419, *p* < .001), vitality (*r* = .313, *p* < .001), working (*r* = .396, *p* < .001), depression (*r* = .202, *p* < .001), memory (*r* = .262, *p* < .001), sleep (*r* = .200, *p* < .001), and happiness (*r* = .135, *p* < .001). Stair climbing showed a strong positive correlation with pain, vitality, and working. Pain showed a positive correlation with vitality (*r* = .288, *p* < .001), working (*r* = .427, *p* < .001), depression (*r* = .308, *p* < .001), memory (*r* = .255, *p* < .001), sleeping (*r* = .311, *p* < .001), and happiness (*r* = .199, *p* < .001). Pain showed a strong positive correlation with working, depression, and sleeping. Vitality showed a positive correlation with work (*r* = .432, *p* < .001), depression (*r* = .353, *p* < .001), memory (*r* = .254, *p* < .001), sleeping (*r* = .332, *p* < .001), and happiness (*r* = .339, *p* < .001). Vitality showed a strong positive correlation with work, depression, sleeping, and happiness. Depression showed a positive correlation with memory (*r* = .299, *p* < .001), sleeping (*r* = .371, *p* < .001), and happiness (*r* = .431, *p* < .001). Depression showed a strong positive correlation with sleeping and happiness. Memory showed positive correlation with sleep (*r* = .245, *p* < .001) and happiness (*r* = .175, *p* < .001). Sleep showed a positive correlation with happiness (*r* = .291, *p* < .001).

### 4.4. Factors Affecting the HINT-Eight

A causal model was established to confirm the effect of physical activity on the QOL. Independent variables were physical activity, age, education level, monthly household income, and grip strength, while the dependent variable was HINT-eight. Stair climbing, pain, vitality, work, depression, memory, sleep, and happiness are all subfactors of the construct idea of QOL. To check whether multicollinearity occurs between variables set by this model, tolerance limits and variance expansion factors were examined. As a result, the tolerance limit value was 0.972~0.710 and the variance expansion factor was 1.408~1.029, suggesting that all models in this study do not have multicollinearity problems (Table 4).

The effect of physical activity on stair climbing was found to be statistically significant in the causal model (Adj. *R*^2^ = .072, *F* = 17.320, *p* < .001). Stair climbing positively affected physical activity, education level, and grip strength: age negatively affected. The effect of physical activity on pain was found to be statistically significant in the causal model (Adj.*R*^2^ = .022, *F* = 5.758, *p* < .001). Pain positively affected as education level and grip strength. The effect of physical activity on vitality was found to be statistically significant in the causal model (Adj.*R*^2^ = .042, *F* = 1.249, *p* < .001). Vitality positively affected physical activity, monthly household income, and grip strength. The effect of physical activity on working was found to be statistically significant in the causal model (Adj.*R*^2^ = .064, *F* = 15.304, *p* < .001). Work positively affected education level, monthly household income, and grip strength, and age negatively affected. The effect of physical activity on depression was found to be statistically significant in the causal model (Adj.*R*^2^ = .006, *F* = 2.339, *p* < .05). Depression positively affected on household income. The effect of physical activity on memory was found to be statistically significant in the causal model (Adj.*R*^2^ = .055, *F* = 13.124, *p* < .001). Memory factors positively affected education level, and age negatively affected. The effect of physical activity on sleeping was found to be statistically significant in the causal model (Adj.*R*^2^ = .028, *F* = 7.010, *p* < .001). Sleep factors positively affected education level, and age negatively affected. The effect of physical activity on happiness was found to be statistically significant in the causal model (Adj.*R*^2^ = .017, *F* = 4.660, *p* < .001). Happiness positively affected physical activity and monthly household income.

## 5. Discussion

In this study, the general characteristics of middle-aged women, differences in physical activity for HINT-eight, and factors affecting HINT-eight were investigated.

Physical activity showed significant differences among general characteristics such as age, economic level, and residence, and among HINT-eight, stairs climbing, vitality, and happiness showed significant differences. In other words, it is similar to the results of previous studies showing that the older the age, the higher the economic level, and the more people live in cities, the more physical activity [36].

The relevance of physical activity was confirmed by classifying the HINT-eight into physical health, social health, mental health, and positive health. The physical health domains were stair climbing, pain, and vitality, and among them, stair climbing, and vitality to be statistically significant. As for the response of the subjects, it that the group without difficulty climbing stairs performed physical activity more than the group with much difficulty. In terms of vitality, it that the group with frequent vitality performed physical activity more than the target group with no vitality at all. Working, a social domain, showed statistically significant results with physical activity. It that the target group, who had no difficulty in working, did more physical activity than the target group who was unable to work. Depression, memory, and sleeping during sleep, which are mental domains, showed statistically significant results with physical activity. It was found that the subjects who had no difficulty in sleeping performed more physical activity than the subjects who could not sleep. The positive domain, happiness, showed statistically significant results with physical activity. In other words, the subjects who were always happy engaged in greater physical activity than the subjects who were unhappy. Through this, it was confirmed that the physical activity of middle-aged women did not have any difficulties in climbing stairs, had vitality, had no difficulty in work, had no difficulty in sleeping, and the happy subjects had more physical activity. Exercise and physical activity have been shown to have a positive effect on QOL [37]. Experimental and cross-sectional studies have shown a positive correlation between the level of physical activity and QOL in healthy individuals [38]. Exercise also reduced depression and enhanced the QOL of inpatients with depression, especially in the physical and mental domains [39].

The QOL in middle-aged means that the individual's sense of happiness or satisfaction should be included in addition to the various objectively observable physical, environmental, economic, and political social indicators, which also represent physical, psychological, social, and spiritual aspects. It also aims to reduce health risk factors of individuals, groups, families, and communities to improve QOL and promote change to a healthy lifestyle. Middle-aged women who maintain close relationships with people around them and receive support do not show depressive tendencies, whereas middle-aged women who have some supporters have more depression [40, 41]. Among the preceding studies related to the QOL of middle-aged women, the relationship between age and QOL among demographic variables is as follows. There have been studies that suggest that age has an effect on happiness [42] and studies that show that life satisfaction grows with age [40]. In this study, age to be related to stair climbing, pain, work, and sleeping among HRQOL subvariables. In other words, as one gets older, it becomes more difficult to undertake physical tasks like climbing stairs and working, the frequency of discomfort rises, and sleeping becomes more difficult, which contradicts previous studies. Furthermore, happiness is not affected by age, showing a difference from previous studies.

Regarding income, Lee [43] said that personal or family income is correlated with the happiness of married women, and that income satisfaction has a greater effect on the QOL than income has a direct effect on the QOL. It was stated that there was a variation in happiness based on income satisfaction. In this study, income level was found to be related to vitality, work, depression, and happiness among HRQOL subvariables. In other words, it was found that as the income level increased, the vitality increased, and the performance in physical activities such as climbing stairs and working was found to be good. This shows similar results to previous studies [43]. As for the educational level and QOL, it has been studied that the higher the education level, the higher the QOL [28]. In this study, education level was related to stair climbing, pain, memory, and happiness among HRQOL subvariables. In other words, that as the level of education increased, the performance of stair climbing physical activities increased, the pain was reduced, and memory and happiness were improved. This shows similar results to previous studies [44].

Depression suggested a major factor that can negatively affect the QOL of middle-aged women. In Korea, 52.3% of middle-aged women experience depression [45], and the incidence of depression is 1.7 to 3 times higher than that of men, and depression occurs mainly in their late 40s [45]. The reason for this high incidence is that it responds specifically to social, economic, and emotional factors that only women experience, and biological differences according to sex [46]. In particular, middle-aged women have more depression and health problems than women who maintain gender equality because they perform household responsibilities and traditional roles [47, 48]. In addition, in a previous study [49], depression was found to be higher in the “lower” income group than in the high-income group and lower in individuals with a spouse than in individuals without a spouse. Another study [50] found a link between low socioeconomic status and high depression and suggested that low and unstable socioeconomic status increases economic stress and promotes negative self-concepts, which in turn lead to depression.

Middle-aged women are manifested in various symptoms. By managing these symptoms in middle-aged women, health can be maintained and promoted in old age, and QOL can be improved [51]. To maintain a healthier and more QOL, middle-aged women need to understand the changes according to the symptoms of middle-aged. In addition, it is important to achieve optimal health by enabling self-care such as activities, exercise management, and dietary management so that they can perform health management on their own.

One of the strengths of this study is that it utilized data from a large population sample. The participants in the KNHANES are a nationally representative sample of civilians in South Korea, and it is possible to generalize results by conducting the analysis according to the guidelines of the KCDC [35, 51]. This study has some limitations. First, because there have not been enough previous studies on middle-aged women, numerous follow-up studies with different factors should be undertaken. Second, although it is possible to extend the interpretation to Korean adults, it would be difficult to extend the interpretation of the results to other countries with cultural differences. Finally, variable extraction was limited because data collected by the government, and not directly collected by the researcher, was used for research.

## 6. Conclusions

In this study, the general characteristics of middle-aged women, differences in physical activity for HINT-eight, and factors affecting HINT-eight were investigated. Physical activity showed significant differences among general characteristics such as age, economic level, and residence, and among HINT-eight, stairs climbing, vitality, and happiness showed significant differences. The physical activity showed a correlation with stair climbing, vitality, and happiness. Stair climbing was correlated with pain, vitality, work, depression, memory, sleep, and happiness. In this study, physical activity was found to be an important influencing factor of HINT-8. Physical activity has been identified as an intervention method that has a positive effect on QOL in previous studies. However, previous studies have identified factors that influence physical activity in general age groups or simply. The greatest significance of this study is that the QOL of middle-aged women through HINT-eight was confirmed and comparatively analyzed from eight specific viewpoints. The results of this study can be usefully used as basic data for establishing a public health strategy by using representative national data to establish strategies for middle-aged women's physical activity and QOL in the future. Considering the differences in the influencing factors revealed through this study, we propose a longitudinal study to verify the effectiveness of strategies to improve the QOL appropriate for each target group.

## Figures and Tables

**Table 1:** Difference in physical activity according to characteristics (*N* = 1,428).

Characteristics	Categories	Physical activity			*x* ^2^	*p*
		No	Yes	Sum		
Age(year)	40s	174 (13.1)	152 (11.5)	326 (24.6)	7.057	0.029
	50s	394 (29.7)	279 (21.0)	673 (50.7)		
	60s	208 (15.7)	119 (9.0)	327 (24.7)		

Marital status	Living together,	632 (47.7)	442 (33.3)	1074 (81.0)	0.404	0.939
	Separated or divorced	75 (5.7)	59 (4.4)	134 (10.1)		
	Widowed	48 (3.6)	34 (2.6)	82 (6.2)		
	Single	21 (1.6)	15 (1.1)	36 (2.7)		

Educational level	≤Elementary school	114 (8.6)	53 (4.0)	167 (12.6)	11.008	0.012
	Middle school	106 (8.0)	62 (4.7)	168 (12.7)		
	High school	337 (25.4)	256 (19.3)	593 (44.8)		
	≥College	218 (16.5)	179 (13.5)	397 (30.0)		

Residential area	Eup and myeon	173 (13.0)	80 (6.0)	253 (19.1)	12.821	0.001
	Dong	603 (45.5)	470 (35.4)	1073 (80.9)		

**Table 2:** The association between HINT-eight and physical activity (*N* = 1,428).

HINT-eight	Subdomain	Categories	Physical activity			*x* ^2^	*p*
			No	Yes	Sum		
Physical health area	Climbing stairs	No difficulty	393 (29.7)	309 (23.4)	702 (53.1)	23.964	0.001
		Some difficulty	314 (23.8)	224 (16.9)	538 (40.7)		
		Lot of difficulty	57 (4.3)	16 (1.2)	73 (5.5)		
		Cannot climb	9 (0.7)	0 (0.0)	9 (0.7)		
	Pain	No pain at all	293 (22.2)	212 (16.0)	505 (38.2)	0.203	0.977
		Slightly present	416 (31.5)	295 (22.3)	711 (53.8)		
		Severe pain	55 (4.2)	36 (2.7)	91 (6.9)		
		Excruciating pain	9 (0.7)	6 (0.5)	15 (1.1)		
	Vitality	Always	225 (17.0)	185 (14.0)	410 (31.0)	20.452	0.001
		Frequently	243 (18.4)	191 (14.5)	434 (32.9)		
		Occasionally	257 (19.5)	162 (12.3)	419 (31.7)		
		Never at all	48 (3.6)	10 (0.8)	58 (4.4)		

Social health area	Work	No difficulty	424 (32.1)	311 (23.5)	735 (55.6)	6.501	0.090
		A little	288 (21.8)	213 (16.1)	501 (37.9)		
		A lot	45 (3.4)	20 (1.5)	65 (4.9)		
		Cannot work	16 (1.2)	5 (0.4)	21 (1.6)		

Mental health area	Depression	Not depressed at all	402 (30.4)	274 (20.7)	676 (51.1)	1.130	0.770
		Often depressed	333 (25.2)	251 (19.0)	584 (44.2)		
		Occasionally depressed	33 (2.5)	20 (1.5)	53 (4.0)		
		Always depressed	5 (0.4)	4 (0.3)	9 (0.7)		
	Memory	No difficulty	339 (25.6)	226 (17.1)	565 (42.7)	4.284	0.232
		A little	409 (30.9)	311 (23.5)	720 (54.5)		
		A lot	23 (1.7)	12 (0.9)	35 (2.6)		
		Never memory	2 (0.2)	0 (0.0)	2 (0.2)		
	Sleep	No difficulty	351 (26.6)	247 (18.7)	598 (45.2)	7.049	0.070
		A little	347 (26.2)	245 (18.5)	592 (44.8)		
		A lot	75 (5.7)	53 (4.0)	128 (9.7)		
		Difficulty sleeping	0 (0.0)	4 (0.3)	4 (0.3)		

Positive health area	Happiness	Always happy	144 (10.9)	110 (8.3)	254 (19.2)	13.300	0.004
		Often happy	261 (19.7)	231 (17.5)	492 (37.2)		
		Occasionally happy	337 (25.5)	190 (14.4)	527 (39.9)		
		Never happy	31 (2.3)	18 (1.4)	49 (3.7)		

**Table 3:** Correlation of HINT-eight and physical activity (*N* = 1,428).

Variable	Physical activity	Climbing stairs	Pain	Vitality	Work	Depression	Memory	Sleep	Happiness
Physical activity	1								
Climbing stairs	.095^∗∗^	1							
Pain	.011	.419^∗∗^	1						
Vitality	.095^∗∗^	.313^∗∗^	.288^∗∗^	1					
Work	.047	.396^∗∗^	.427^∗∗^	.432^∗∗^	1				
Depression	-.013	.202^∗∗^	.308^∗∗^	.353^∗∗^	.369^∗∗^	1			
Memory	-.012	.262^∗∗^	.255^∗∗^	.254^∗∗^	.317^∗∗^	.299^∗∗^	1		
Sleep	-.014	.200^∗∗^	.311^∗∗^	.332^∗∗^	.349^∗∗^	.371^∗∗^	.245^∗∗^	1	
Happiness	.072^∗∗^	.135^∗∗^	.199^∗∗^	.339^∗∗^	.261^∗∗^	.431^∗∗^	.175^∗∗^	.291^∗∗^	1

^∗^ *p* < 0.05 and^∗∗^*p* < 0.001.

**Table 4:** Factors affecting the HINT-eight (*N* = 1,428).

Variable		Nonstandardized coefficients		Standardization coefficient	*t*	*p*	Model fitness
Dependent	Independent	*B*	SE	*β*			
(1) Stair climbing	Constant	3.679	.237		15.500	<.001	*R* ^2^ = .044Adj.*R*^2^ = .072*F* = 17.320*p* < .001
	Physical activity	.069	.035	.055	2.009	<.05	
	Age	-.015	.003	-.144	-4.713	<.001	
	Education level	.022	.006	.116	3.606	<.001	
	Household income	.000	.000	.036	1.244	.214	
	Grip	.014	.004	.093	3.368	<.001	

(2) Pain	Constant	3.151	.251		12.545	<.001	*R* ^2^ = .027Adj.*R*^2^ = .022*F* = 5.758*p* < .001
	Physical activity	-.005	.037	-.004	-.133	.894	
	Age	-.006	.003	-.058	-1.845	<.10	
	Education level	.018	.007	.092	2.783	<.01	
	Household income	.000	.000	.012	.405	.686	
	Grip	.012	.004	.080	2.817	<.01	

(3) Vitality	Constant	1.949	.347		5.621	<.001	*R* ^2^ = .047Adj.*R*^2^ = .042*F* = 10.249*p* < .001
	Physical activity	.111	.050	.062	2.198	<.05	
	Age	-.001	.005	-.005	-.145	.885	
	Education level	.013	.009	.048	1.481	.139	
	Household income	.000	.000	.097	3.259	<.001	
	Grip	.027	.006	.127	4.509	<.001	

(4) Working	Constant	3.328	.253		12.825	<.001	*R* ^2^ = .068Adj.*R*^2^ = .064*F* = 15.304*p* < .001
	Physical activity	.016	.037	.012	.435	.663	
	Age	-.008	.003	-.075	-2.435	<.05	
	Education level	.025	.007	.123	3.790	<.001	
	Household income	.000	.000	.110	3.724	<.001	
	Grip	.014	.004	.088	3.187	<.001	

(5) Depression	Constant	3.357	.239		14.072	<.001	*R* ^2^ = .000Adj.*R*^2^ = .006*F* = 2.339*p* < .05
	Physical activity	-.025	.035	-.020	-.715	.475	
	Age	-.003	.003	-.024	-.767	.444	
	Education level	.007	.006	.038	1.141	.254	
	Household income	.000	.000	.060	1.987	<.05	
	Grip	.004	.004	.026	.916	.360	

(6) Memory	Constant	3.588	.212		16.906	<.001	*R* ^2^ = .059Adj.*R*^2^ = .055*F* = 13.124*p* < .001
	Physical activity	-.038	.031	-.034	-1.241	.215	
	Age	-.011	.003	-.117	-3.811	.001	
	Education level	.025	.006	.148	4.551	.001	
	Residence	.006	.039	.004	.148	.882	
	Household income	.000	.000	.025	.840	.401	
	Grip	.005	.004	.035	1.249	.212	

(7) Sleeping	Constant	3.752	.258		14.517	<.001	*R* ^2^ = .032Adj.*R*^2^ = .028*F* = 7.010*p* < .001
	Physical activity	-.029	.038	-.022	-.772	.440	
	Age	-.011	.004	-.094	-3.023	<.01	
	Education level	.019	.007	.092	2.797	<.01	
	Household income	.000	.000	.048	1.609	.108	
	Grip	-.004	.004	-.025	-.900	.368	

(8) Happiness	Constant	2.522	.318		8.028	<.001	*R* ^2^ = .022Adj.*R*^2^ = .017*F* = 4.660*p* < .001
	Physical activity	.127	.046	.078	2.738	<.01	
	Age	-.002	.004	-.014	-.434	.665	
	Education level	-.004	.008	-.017	-.512	.609	
	Household income	.000	.000	.112	3.714	<.001	
	Grip	.005	.006	.025	.893	.372	

## Data Availability

KNHANES data are publicly accessible. The data can be accessed and downloaded from the KNHANES homepage (URL: https://knhanes.kdca.go.kr/knhanes/eng/index.do).
